RETRACTED

# Synergistic Effect of Zuo Jin Wan on DDP-Induced Apoptosis in Human Gastric Cancer SGC-7901/DDP Cells

**DOI:** 10.1155/2014/724764

**Published:** 2014-03-03

**Authors:** Qing-Feng Tang, Qing Ji, Yan-Yan Qiu, Ai-Li Cao, Yang-Feng Chi, Bo Liang, Wen Peng, Pei-Hao Yin

**Affiliations:** ^1^Department of Clinical Laboratories & Experimental Center, Putuo Hospital, Shanghai University of Traditional Chinese Medicine, Shanghai 200062, China; ^2^Department of General Surgery, Putuo Hospital, Shanghai University of Traditional Chinese Medicine, Shanghai 200062, China; ^3^Department of Nephrology, Putuo Hospital, Shanghai University of Traditional Chinese Medicine, Shanghai 200062, China

## Abstract

A traditional Chinese medicine (TCM) formula, Zuo Jin Wan (ZJW), has been found as an anticancer drug in human cancer. In this study, we investigated the synergistic effect of ZJW extracts on DDP-induced apoptosis in human gastric cancer SGC-7901/DDP cells. Our results demonstrated that ZJW extracts could increase the sensitivity of SGC-7901/DDP cells to DDP by increasing the concentration of DDP in cytoplasm and enhance the proapoptosis of DDP by upregulating the JNK and Bax expression, downregulating the Bcl-2 expression, increasing the accumulation of Cytochrome C in cytoplasm, and promoting the activities of caspase-3 and caspase-9. *In vivo*, ZJW extracts enhanced the inhibiting effect of DDP on tumor growth in SGC-7901/DDP xenograft model and upregulated the expression of p-JNK and Bax but downregulated the Bcl-2 expression in xenograft tumors. In conclusion, *in vitro* and *in vivo*, ZJW extracts could enhance the proapoptotic effect of DDP by promoting the activation of JNK and the expression of Bcl-2, inhibiting the Bax expression, followed by increasing the release of Cytochrome C from mitochondria to cytoplasm, and finally activating the caspase cade reaction. Our results implied that ZJW might serve as a synergistic drug with chemotherapeutic drugs DDP in the treatment of gastric cancer.

## 1. Introduction

Presently, chemotherapeutic drug resistance has been recognized as one of the primary problems in the therapy of cancer [1–3]. Because of its complicated mechanism, effective methods for solving this problem still have not been found. As far as we know, Traditional Chinese Medicines (TCMs) have been used as western medicines or health supplements in the past thousands of years. In clinical practice, lots of Traditional Chinese prescriptions and formulate, which are based on TCM principles, have been identified as effective anticancer drugs in cancer patients, such as gastric cancer [4], breast carcinoma [5], and colorectal cancer [6]. Compared with chemotherapeutic drugs, Traditional Chinese Medicines could also control cancer progression effectively [7], prolong survival periods [8], and improve life quality [9].

RETRACTED

Zuo Jin Wan (ZJW) is a typical TCM formula, which consists of the Rhizoma Coptidis and Fructus Evodiae in the ratio of 6 : 1 (w/w). Fructus Evodiae could induce apoptosis in cancer cells, such as human hepatocellular carcinoma SMMC-7721 cells [10], human melanoma A375-S2 cells [11], and human colorectal carcinoma COLO-205 cells [12]. Since ZJW herbal formula has anticancer effect, its underlying mechanisms need further investigation. In the present study, we elucidated the effect and the molecular mechanism of Chinese herbs formula ZJW in human gastric cancer SGC-7901/DDP cells *in vitro* and* in vivo* and provided possible target for the therapy of gastric cancer.

## 2. Materials and Methods

### 2.1. Preparation of the ZJW Extracts

ZJW was formulated by Rhizoma Coptidis and Evodiae, in a ratio of 6 : 1. The above two herbs were purchased from Putuo Hospital, Shanghai University of Traditional Chinese Medicine. ZJW was extracted twice by refluxing in ethanol (1 : 8, v/v), each time for 1 hour. Put together the extracted mixtures were filtrated, concentrated, and dried in vacuum at 60°C. The yield of dried powder was about 24.4%, and the extract was stored at 4°C. Preparation of the ZJW extracts was standardized and quality controlled according to the guidelines from Chinese State Food and Drug Administration (SFDA). For all the experiment, the above ZJW extract powders were dissolved in RPMI 1640 medium by vortex, ultrasonic, and bath, followed by filtration, and formulated into a solution of desired concentration.

### 2.2. Cell Culture

SGC-7901/DDP cell lines were obtained from Keygen Biotech Co., Ltd. (Nanjing, China). The cells were grown in RPMI 1640 medium supplemented with 10% (v/v) fetal calf serum (FCS, Gibico, USA), 100 *μ*g/mL streptomycin, and 100 units/mL penicillin, in 5% CO_2_ humidified atmosphere, at 37°C. SGC-7901/DDP cells were routinely maintained in the above RPMI 1640 medium containing 10 *μ*g/mL Diamminedichloroplatinum (DDP, Qilu Pharmaceutical Co., Ltd., Shandong, China).

### 2.3. Analysis of Cells Viability

Cell Counting Kit-8 (CCK-8) was chosen to determine cells proliferation. Briefly, SGC-7901/DDP cells were seeded in 96-well plates at 1 × 10^4^ cells/well; when the cells reached 60% confluence, the medium was removed and replaced with fresh medium containing varying concentrations of ZJW and incubated for 48 hours. After incubation with culture medium containing CCK-8 reagent for 4 hours, the absorbance was detected at 450 nm using a microplate reader (Biorad, USA). All the experiments were repeated three times.

RETRACTED

### 2.4. ICP-MS Analysis

SGC-7901/DDP cells were washed three times with PBS and digested, and the collected cells were washed. 500 *μ*L ddH_2_O was added and the cells were broken by freezing and thawing with liquid nitrogen repeatedly followed by sonication. They were centrifuged for 10 min at 14000 rpm/min, the supernatant was collected, dried under vacuum for 24 h, and dissolved in PBS. The dissolved samples were digested by 2 mL nitric acid followed by 1 mL perchloric acid, cooled down, set to constant volume of 10 mL, and ultrafiltrated. The ultrafiltrated samples (10 mL) were diluted using a Gilson ASPEC XLi programme to deliver 1.8 mL of iridium internal standard (0.005 mg/mL, in 1% nitric acid) and mixed thoroughly. Intracellular accumulation of DDP in each sample was determined by ultrasensitive multicollector inductively coupled with mass spectrometry (ICP-MS) as previously described [13].

### 2.5. Flow Cytometry Analysis

SGC-7901/DDP cells were plated in 6-well plates at 4 × 10^5^ cells/well and starved overnight in RPMI 1640 medium with 0.5% serum. Being treated with ZJW of different concentration for 48 hours, the cells were collected, washed with cold PBS twice, and resuspended gently in 400 *μ*L binding buffer. 5 *μ*L Annexin V-FITC was added to the above cells solution, gently vortexed, and incubated for 10 min at 4°C avoiding the light. 10 *μ*L propidium iodide (PI) was added and cultured for another 5 minutes. Flow cytometry was then conducted using FACSCalibur Flow Cytometry (BD Biosciences, USA), and the results were analyzed with CellQuest software.

### 2.6. Western Blotting

Cytoplasmic proteins from SGC-7901/DDP cells were prepared using a ProteoJET cytoplasmic kit (Fermentas, USA). All proteins were loaded onto SDS-PAGE gels for electrophoresis, transferred onto PVDF membranes, and blocked in 5% BSA prior to incubation with primary and secondary antibody. The resulting immunocomplexes were visualized by enhanced chemiluminescence. Each lane was photographed and quantified. All the experiments were repeated three times.

### 2.7. Analysis of Caspase-3 and Caspase-9 Protease Activity

SGC-7901/DDP cells were seeded in a 96-well plate and starved overnight in RPMI 1640 medium with 0.5% serum. Being treated with ZJW of different concentration for 48 hours, 100 *μ*L of Caspase-Glo 3 or Caspase-Glo 9 reagent (Promega, USA) was added to each sample and incubated at room temperature for another 2 hours. The luciferase activity was measured using a TD 20/20 luminometer (Promega, USA). Each sample was measured in triplicate.

### 2.8. Tumor Mouse Model

SGC-7901/DDP cells were harvested in serum-free PBS and 100 *μ*L single-cell suspensions (2 × 10^7^ cells/mL) were injected into the subcutaneous area of female BALB/c nude mice (4–6 weeks old, SLAC Laboratory Lab, Shanghai, China). When the tumors reached an average size of 100 mm^3^, the mice were randomized into 5 groups (*n* = 10). Mice in group 1 were administered with normal saline daily, mice in group 2 were administered with 10 *μ*g/mL DDP, mice in groups 3, 4, and 5 proceeded intragastric administration of ZJW extracts at doses of different concentration (dose calculation is referred in our previous experiment [14]), plus 10 *μ*g/mL DDP, respectively. The length and width of tumors were recorded every 7 days. After 35 days, animals were sacrificed by cervical dislocation in deep anesthesia of CO_2_ and primary tumors were surgically removed and weighed. Tumor sizes were evaluated using the formula: length × width^2^ × 0.52. The primary tumors were analyzed by hematoxylin-eosin (HE) staining, and p-JNK, Bax, and Bcl-2 proteins were detected by immunohistochemistry. All experimental protocols were reviewed and approved by the Committee on Animal Experimentation.

RETRACTED

### 2.9. Statistical Analysis

The data processing was performed with SPSS18 Software. All the data results are expressed as mean ± standard deviation $\left(\overset{-}{X}\pm S\right)$. The mean values of two groups were compared by Student's *t* test. A value of *P* < 0.05 was statistically significant.

## 3. Results

### 3.1. Effect of ZJW Extracts on the Sensitivity to DDP in SGC-7901/DDP Cells

Our previous research has made quantitative analysis of various active compounds in the ZJW extracts [14]. Simply, quantitative results of jatrorrhizine, palmatine, and berberine in Rhizoma Coptidis were 3.8%, 6.4%, and 57.1%, respectively; evodiamine and rutaecarpine in Evodia were 2.29% and 3.18%.

For avoiding the possibility that inhibition of cell proliferation is due to cytotoxicity, the cytotoxic concentration of ZJW extracts on SGC-7901/DDP cells was investigated first by CCK-8 assay. At present, IC10 was a permitted standardization of the noncytotoxic dose, and our study showed that the IC10 of ZJW extracts on SGC-7901/DDP cells was about 50 *μ*g/mL (Figure 1(a)). Next, to determine the best effect of ZJW on the sensitivity to DDP in SGC-7901/DDP cells, IC50 of DDP on SGC-7901/DDP cells treated or no treated with 50 *μ*g/mL ZJW extracts was detected. The results showed that IC50 of DDP on lonely SGC-7901/DDP cells was 6.73 ± 0.72 *μ*g/mL, but with addition of 50 *μ*g/mL ZJW extracts, IC50 of DDP decreased from 6.73 ± 0.72 *μ*g/mL to 2.83 ± 0.41 *μ*g/mL (Figure 1(b)). Finally, we analyzed the effect of ZJW extracts with different concentrations on SGC-7901/DDP cells, in the presence of 6.73 ± 0.72 *μ*g/mL DDP. Data showed that ZJW extracts could enhance the sensitivity of DDP on SGC-7901/DDP cells in a dose dependent manner (Figure 1(c)).

RETRACTED

### 3.2. Effect of ZJW Extracts on the Apoptosis and Cycle of SGC-7901/DDP Cells

Flow cytometry was performed to see the effect of ZJW extracts on the apoptosis and cycle of SGC-7901/DDP cells. The results showed that exposure to ZJW extracts increased DDP-induced cell apoptosis in a dose dependent manner (Figure 2(a)). However, cell cycle analysis showed that there was little change in any phase arrest in response to treatment with ZJW extracts compared with control group (Figure 2(b)). This suggested that ZJW extracts did not change cell cycle in SGC-7901/DDP cells, and the effect of ZJW extracts was most likely obtained by enhancing the DDP-induced apoptosis.

### 3.3. Impact of ZJW Extracts on the Accumulation of DDP in SGC-7901/DDP Cells

Using ICP-MS for determination of the changed intracellular DDP concentration in SGC-7901/DDP cells, we found that, with 6.73 *μ*g/mL DDP and different concentrations of ZJW extracts exposed to SGC-7901/DDP cells for 48 hours, the intracellular accumulation of DDP increased in a dose dependent manner (Figure 3). This implied that ZJW extracts had the function of promoting translocation of DDP from extracellular to intracellular.

### 3.4. Effect of ZJW Extracts on the Apoptosis-Related Proteins in SGC-7901/DDP Cells

To further investigate the underlying proapoptotic mechanisms of ZJW extracts on SGC-7901/DDP cells, we detected the levels of apoptosis-related proteins in SGC-7901/DDP cells, including JNK, p-JNK, Bax, Bcl-2, Cytochrome C, Caspase-9, and Caspase-3. As shown in Figures 4(a) and 4(b), with the increasing concentration of ZJW extracts, 12.5 *μ*g/mL, 25 *μ*g/mL, and 50 *μ*g/mL, the active level of p-JNK was significantly increased in SGC-7901/DDP cells, although the total JNK protein expression changed a little. In addition, the expression of Bax and Cytochrome C increased but Bcl-2 decreased in a dose dependent manner. The activities of Caspase-9 and Caspase-3 were also detected, and their activities elevated with the increasing concentration of ZJW extracts (Figure 4(c)). This suggested that the proapoptotic effect of ZJW extracts in SGC-7901/DDP cells might be dependent on the activation of JNK, followed by the promotion of Bcl-2 and inhibition of Bax, further increased release of Cytochrome C from mitochondria to cytoplasm, and finally the activation of caspase cade reaction.

### 3.5. Impact of ZJW Extracts on Subcutaneous Xenograft of SGC-7901/DDP in Nude Mice

To explore whether ZJW extracts enhanced the proapoptotic effect of DDP *in vivo*, we employed a subcutaneous xenograft model. As shown in Figure 5(a), the combination of DDP and ZJW extracts produced a significant inhibition of tumor growth compared with animals treated with DDP alone, and ZJW extracts helped DDP inhibit the mice tumor volume in a dose dependent manner. The final tumor weights also showed the synergistic effect ZJW extracts and DDP (Figure 5(b)).

RETRACTED

By HE staining of tumor tissues, we observed the morphological changes of tumor cells by inverted microscope. In the SGC-7901/DDP group, tumor cells were arranged regularly, growth of tumor cells was active, more mitosis, and less cytoplasm. In the 0.6 mg/kg DDP alone group, very small necrosis appeared, and the volume of tumor cells became smaller. In the presence of 0.6 mg/kg DDP, with the increasing concentration of ZJW extracts, the necrosis area of tumor sheet increased by degrees, cells became more and more smaller and were arranged more irregularly, the nuclei was dark stained and condensed, and rich cytoplasm and a piece of hyaline change were seen (Figure 5(c)).

Additionally, we detected the expression of p-JNK, Bax, and Bcl-2 in the xenograft tumor tissues by immunohistochemistry. The pictures showed that the expression of p-JNK and Bax increased with the gradually increasing concentration of ZJW extracts. However, expression of Bcl-2 was the opposite trend. This implied that ZJW extracts might enhance the proapoptotic effect of DDP and could be provided as synergistic chemotherapy drugs with DDP in the treatment of gastric cancer (Figure 6).

## 4. Discussions

In the process of cancer chemotherapy, the most intractable problem is the appearance of drug resistance of tumor cells to chemotherapeutic agents. In clinical practice, Chinese medicine drugs have showed good synergism in chemotherapy, which have been proven in numerous studies [6, 15, 16]. Chinese medicine believes that one of the pathogenesis of gastric cancer is the disharmony of liver and gastric, so there was the strong theoretical basis on the ZJW treatment of gastric cancer from the perspective of pathogenesis. In recent years, ZJW showed comprehensive potentiality in early prevention and treatment of cancer [10–12]. ZJW could inhibit acquired multidrug resistance of tumor originated from S180 cells and improve the quality life, body mass, white blood cell count, and immune organs index of tumor-bearing mice [17]. Modern pharmacological studies have shown that the compatibility of two drugs could be used to inhibit the growth and migration of tumor cells, promote apoptosis of tumor cells, and block the effect of cancer-promoting substances on potential cancer cells [18, 19].

RETRACTED

To further investigate the effect mechanism of ZJW extracts on gastric cancer, human gastric cancer SGC-7901/DDP cells, which have resistance to a variety of chemotherapeutic drugs, were chosen for our present study. Immediately we determined the nontoxic dose of ZJW extracts, combined ZJW extracts with DDP to treat SGC-7901/DDP cells, and found that ZJW extracts could increase the killing effect of DDP on SGC-7901/DDP cells and elevate the apoptosis rate of SGC-7901/DDP cells. However, ZJW extracts had little effect on the cycle of SGC-7901/DDP cells. Further research demonstrated that ZJW extracts made an increasing accumulation of DDP in SGC-7901/DDP cells, which implied that ZJW extracts had the function of promoting translocation of DDP from extracellular to intracellular.

While investigating the underlying proapoptotic mechanisms of ZJW extracts on DDP-induced apoptosis in SGC-7901/DDP cells, we found that the synergistic effect of ZJW extracts on proapoptosis of DDP in SGC-7901/DDP cells might be dependent on the activation of JNK, which played vital role in the development of cancer [20, 21]. Upon activation of JNK, the p-JNK blocked the Bax level and promoted the Bcl-2 level. As we have known, the ratio of Bax and Bcl-2 was responsible for a variety process of apoptosis [22–24]. Hereafter, we found that release of Cytochrome C from mitochondria to cytoplasm increased, which involved in typically mitochondrial apoptosis pathway [25, 26]. Finally, caspase-9 and caspase-3 were activated, which led to the ultimate apoptosis of cancer cells [27, 28]. According to *in vitro* results, we conducted subcutaneous xenograft model to validate the possible synergistic effect of ZJW extracts on proapoptosis of DDP *in vivo*.

In light of our *in vitro* data on the effect of ZJW extracts in human gastric cancer SGC-7901/DDP cells to chemotherapeutic drugs, we examined the *in vivo* therapeutic potential of ZJW extracts. *In vivo* experiments results showed that the anticancer effect of ZJW extracts on SGC-7901/DDP cells xenograft was better than that of DDP alone group. In this study, we provided evidence that combination of DDP with herbal medicine formula ZJW extracts promoted the growth inhibition effect of xenograft tumors and promoted the apoptosis of tumor cells in xenograft tumors. The immunohistochemistry results showed that the expression of p-JNK and Bax increased, but Bcl-2 decreased with the gradually increasing concentration of ZJW extracts, which implied that ZJW extracts might enhance the proapoptotic effect of DDP and could be provided as synergistic drugs with DDP in the treatment of gastric cancer.

RETRACTED

In conclusion, noncytotoxic ZJW extracts could enhance the proapoptotic effect of DDP in human gastric cancer SGC-7901/DDP cells through increasing the intracellular accumulation of DDP, which promoted the activation of JNK, followed by the promotion of Bcl-2 and inhibition of Bax, further increased release of Cytochrome C from mitochondria to cytoplasm, and finally the activation of caspase cade reaction.

## Figures and Tables

**Figure 1:** Effect of ZJW extracts on the sensitivity to chemotherapeutic drug in SGC-7901/DDP cells. (a) Cells were treated with ZJW extracts of gradual concentrations for 48 hours, and cell survival proportion was analyzed by CCK-8 assay. (b) Effect of DDP on the proliferation of SGC-7901/DDP cells treated with or without 50 *μ*g/mL ZJW extracts for 48 hours was performed by CCK-8 assay. (c) CCK-8 assay was used to detect IC50 of DDP in SGC-7901/DDP cells treated with ZJW extracts of 12.5 *μ*g/mL, 25 *μ*g/mL, and 50 *μ*g/mL for 48 h. *P < 0.05 or **P < 0.01, versus control groups treated without ZJW extracts.

**Figure 2:** Effect of ZJW extracts on the apoptosis and cycle of SGC-7901/DDP cells. (a), (b) Flow cytometry analysis of cell apoptosis and cycle distribution was performed on SGC-7901/DDP cells treated, respectively, with 6.73 *μ*g/mL DDP, 6.73 *μ*g/mL DDP + 12.5 *μ*g/mL ZJW, 6.73 *μ*g/mL DDP + 25 *μ*g/mL ZJW, and 6.73 *μ*g/mL DDP + 50 *μ*g/mL ZJW, with the control group treated without DDP and ZJW.

**Figure 3:** Impact of ZJW extracts on the accumulation of DDP in SGC-7901/DDP cells. ICP-MS method was used to detect intracellular DDP accumulation in SGC-7901/DDP cells treated with ZJW extracts of 12.5 *μ*g/mL, 25 *μ*g/mL, and 50 *μ*g/mL for 48 h. *P < 0.05 or **P < 0.01, in contrast to control groups treated without ZJW extracts.

**Figure 4:** Effect of ZJW extracts on the apoptosis-related proteins in SGC-7901/DDP cells. (a) Western blotting was carried out to detect the expression level of total JNK, p-JNK, Bax, Bcl-2, and Cytochrome C in SGC-7901/DDP cells treated with ZJW extracts of 12.5 *μ*g/mL, 25 *μ*g/mL, and 50 *μ*g/mL for 48 h. GAPDH was used as internal reference. (b) Quantity of the expression level of total JNK, p-JNK, Bax, Bcl-2, and Cytochrome C was performed, *P < 0.05 or **P < 0.01, in contrast to control groups treated with DDP alone. (c) Activities of caspase-9 and caspase-3 were detected in SGC-7901/DDP cells treated with ZJW extracts of 12.5 *μ*g/mL, 25 *μ*g/mL, and 50 *μ*g/mL for 48 h. *P < 0.05 or **P < 0.01, in contrast to groups treated with DDP alone.

**Figure 5:** Impact of ZJW extracts on subcutaneous xenograft of SGC-7901/DDP cells in nude mice. (a) Mice were divided into five groups, group 1: normal saline; group 2: 5 mg/kg DDP; group 3: 500 mg/kg ZJW (L-dose) + 0.6 mg/kg DDP; group 4: 1000 mg/kg ZJW (M-dose) + 0.6 mg/kg DDP; group 5: 2000 mg/kg ZJW (H-dose) + 0.6 mg/kg DDP. Tumor volume was measured every seven days. (b) Tumors were surgically removed from nude mice and weighed after administration for 35 days. *P < 0.05 or **P < 0.01, in contrast to groups treated with DDP alone. (c) Morphological changes of tumor cells were detected by HE staining, and the photograph was observed by inverted microscope.

RETRACTED

**Figure 6:** Impact of ZJW extracts on the expression level of p-JNK, Bax, and Bcl-2 *in vivo*. The xenograft tumor tissues in mice of all groups was subjected to immunohistochemistry analysis using antibody of p-JNK, Bax, and Bcl-2, and the pictures were magnified ×200 in microscope.
